The article "The rs13347 Polymorphism of the CD44 Gene Is Associated with the Risk of Kidney Stones Disease in the Chinese Han Population of Northeast Sichuan, China" was retracted in 2023. Reasons: signs of a paper mill; compromised peer review; unreliable results or conclusions.

# The rs13347 Polymorphism of the CD44 Gene Is Associated with the Risk of Kidney Stones Disease in the Chinese Han Population of Northeast Sichuan, China

**DOI:** 10.1155/2022/6481260

**Published:** 2022-01-13

**Authors:** Qiao Ying, Guixi Liu, Wenjun Zhou, Jianhua Lan, Jianhui Du, Xianfu Tang, Xiaohan Xu

**Affiliations:** ^1^Department of Urology, People's Hospital of Guang'an City (West China-Guang'an Hospital, Sichuan University), No.1, Section 4, Binhe Road, Guang'an District, Guang'an City, Sichuan Province 638000, China; ^2^Department of Urology, The Third Hospital of Mianyang (Sichuan Mental Health Center), No. 190, East Section of Jiannan Road, Mianyang City, Sichuan Province 621000, China

## Abstract

**Objective:**

To investigate the association between the rs13347 polymorphism of the CD44 gene and the risk of kidney stone disease (KSD) in the Han population of northeast Sichuan, China, so as to provide a theoretical basis for the treatment of KSD.

**Methods:**

We used PCR-restriction fragment length polymorphism (RFLP) technique to perform genotyping at rs13347 locus of the CD44 gene in the KSD group and the gontrol group. SNP Hardy-Weinberg equilibrium (HWE) testing was used to confirm the balance of genetic inheritance. Multivariate logistic regression analysis was used for the assessment of rs13347 polymorphism and the risk of developing KSD and to compare the relationship between the polymorphism of rs13347 and clinical characteristics of patients with KSD.

**Results:**

Genotypic results of rs13347 locus of the CD44 gene in the two groups were consistent with the SNP-HWE test, indicating the genetic balance. At the same time, multivariate logistic regression analysis indicated that subjects with CT and TT genotypes at rs13347 in the CD44 gene were more likely to have KSD, and there was a higher prevalence rate in males. Furthermore, carrying allele T at rs13347 was also a risk factor for KSD. In addition, people carrying CT and TT genotypes at rs13347 also have a significantly increased risk of relapsing KSD.

**Conclusion:**

The rs13347 polymorphism of the CD44 gene may be associated with the risk of KSD in the Han population of northeast Sichuan in China, and the recurrence rate of KSD in the carriers of CT and TT genotypes is higher.

## 1. Introduction

Kidney stone disease (KSD), one of the most common urological diseases, is a disease formed due to the abnormal accumulation of crystalline material in the kidney, which can lead to renal impairment, urinary tract obstruction, infection and other diseases [1]. According to statistics, the global incidence of KSD is 3-5%, which has affected the normal life of 15% of the global population, and the prevalence rate and incidence are increasing year by year [2]. In recent years, the incidence of KSD in China has also shown a rising trend and China has been one of the highest incidence areas in the world [3]. The incidence of KSD is regional, with approximately 7% in Europe, 3% in Asia, and 15% in North America [4]. In China, KSD is more common in areas south of the Yangtze River, with an incidence as high as 7.5% [3]. It has been shown that the occurrence of KSD is related to factors such as genes, dietary habits, environment and metabolism [4]. At present, there are two main ways to treat KSD: for patients with stones less than 5 mm in diameter and without urinary tract obstruction or infection, diet adjustment and drug treatment can be used to control the development of stones; for patients who failed to respond to drug treatment, surgical methods can be used to clean stones, such as shock wave lithotripsy, ureteroscopic lithotripsy, percutaneous nephrolithotomy and laparoscopic ureterolithotomy. Although there are many methods to treat KSD, some studies have pointed out that the postoperative recurrence rate of KSD patients can reach up to 28-52%, seriously affecting the quality of patients' life [5]. Therefore, in-depth study of the pathogenesis of KSD is of great significance for the treatment and prevention of its occurrence.

The article "The rs13347 Polymorphism of the CD44 Gene Is Associated with the Risk of Kidney Stones Disease in the Chinese Han Population of Northeast Sichuan, China" was retracted in 2023. Reasons: signs of a paper mill; compromised peer review; unreliable results or conclusions.

CD44 is a type of cell adhesion factor and a ubiquitous multifunctional transmembrane glycoprotein [6]. Initial studies revealed that CD44 is associated with homing of lymphocytes, so it is also known as lymphocyte homing receptor [7]. In recent years, it has been shown that CD44 is not only involved in the regulation of the growth and metastasis process of tumor cells, but also a key molecule in the transmission of information between cells, playing an important role in maintaining the homeostasis of the intracellular environment and the integrity of the extracellular matrix [8]. On the one hand, CD44 is one of the major receptors for osteopontin (OPN) [6]. It has been shown that OPN can regulate the function of cells, cell adhesion, and participate in the repair process after kidney tissue injury after mutual binding with CD44 [9, 10]. In addition, the signals transmitted after OPN binds to CD44 can mediate a series of cellular and intercellular reactions, which leads to chemotactic movement of macrophages that gobbled up stone and crystals, and this reaction is also an important factor in the formation of kidney stones [11]. On the other hand, CD44 is produced by alternative splicing of mutant exons and exists in a variety of subtypes [12]. Recent studies have shown that the polymorphism of CD44 is associated with the risk of developing a variety of cancers, including breast cancer [13], gastric cancer [14] and colorectal cancer [15]. Jiang et al. pointed out that when the rs13347 locus of the CD44 gene is changed from the most common CC genotype to the CT or TT genotype, it increases the probability that an individual has breast cancer [16]. In addition, Wu et al. found that when CC genotype in rs13347 was changed into T genotypes (CT and TT), the binding site of miR-503-3p was destroyed, which resulted in an increased expression of CD44 and an increased incidence of colorectal cancer [17]. From this, it can be obtained that the conventional expression of the CD44 gene is related to the adhesion and aggregation of cells, while the polymorphism at rs13347 is related to the abnormal expression of the CD44 gene. But there are few reports on the association between polymorphisms at rs13347 in the CD44 gene and the development of KSD. Therefore, this study was performed to investigate the relationship between rs13347 polymorphism of the CD44 gene and the risk of KSD in the Han population of northeast Sichuan in China, and for the purpose of providing a theoretical basis for the in-depth study of the pathogenesis of KSD.

The article "The rs13347 Polymorphism of the CD44 Gene Is Associated with the Risk of Kidney Stones Disease in the Chinese Han Population of Northeast Sichuan, China" was retracted in 2023. Reasons: signs of a paper mill; compromised peer review; unreliable results or conclusions.

## 2. Materials and Methods

### 2.1. Study Subjects

A total of 100 kidney stone disease (KSD) patients who were diagnosed in our hospital from June 2017 to December 2019 were collected as the experimental group (KSD group), and 124 healthy individuals who underwent physical examination in our hospital during the same period were collected as the control group (Control group). All patients in this study gave informed consent to the study and signed an informed consent form. This study was approved by the Clinical Experimental Ethics Committee of our hospital and strictly followed the Declaration of Helsinki.

Inclusion criteria are as follows: (1) all subjects were unrelated Han population from the northeast area of Sichuan in China and (2) all patients were diagnosed with KSD by ultrasound or X-ray examination.

Exclusion criteria are as follows: (1) secondary KSD caused by urethral obstruction, hyperparathyroidism, and other factors; (2) history of renal tubular acidosis; (3) patients with renal failure, gout, sponge kidney, vitamin D poisoning, or hyperuricemia; (4) patients suffered from adrenal disease and pituitary tumor; (5) patients with chronic liver and intestinal diseases; and (6) patients with concurrent tumors.

### 2.2. Collection of Basic Data of Subjects

The contents of data collection included age, gender, BMI, alcoholism, diabetes, hypertension, hyperlipidemia, and recurrent KSD.

### 2.3. Polymerase Chain Reaction-Restriction Fragment Length Polymorphism

Genomic DNA was extracted using a whole-blood DNA extraction kit (Sangon Biotech, Shanghai), and the concentration was determined by a nucleic acid quantitative instrument (Thermo, USA). PCR amplification was performed according to the instruction of PCR fluorescence kit (Takala, Japan), and the reaction conditions were 95° C for 10 min, 95° C for 15 s, 60° C for 30 s, and 72° C for 45 s, 40 cycles were performed. Later, the amplified products were digested by MspI endonuclease (BioLabs, Singapore) for 16 hours in a 37° C water bath. Afterwards, electrophoresis was performed with 2% gel, and the digestion results were observed in a gel imager (Bio-rad, USA). Primer sequences, rs13347: F: 5′-ACGATAGAAATAAGGGAGG-3′; R: 5′-GCAAGGGTTTGTGAAGAC-3′.

The article "The rs13347 Polymorphism of the CD44 Gene Is Associated with the Risk of Kidney Stones Disease in the Chinese Han Population of Northeast Sichuan, China" was retracted in 2023. Reasons: signs of a paper mill; compromised peer review; unreliable results or conclusions.

### 2.4. Statistical Analysis

Data were statistically processed using SPSS 21.0. Enumeration data were described by number of cases and percentage (%) and analyzed by chi-square test. Measurement data were expressed as mean ± standard deviation (SD), and pairwise comparisons were performed using two independent samples t-test. Hardy-Weinberg equilibrium (HWE) was performed in two groups of subjects to detect the genotype distribution of the rs187115 and rs13347 polymorphisms in CD44 using *χ*^2^ statistics [18]. Multivariate logistic regression analysis was performed to assess the risk of rs13347 polymorphism and the occurrence of KSD, and odds ratio (OR) and 95% confidence interval (CI) indicated the strength of association. *p* < 0.05 was considered to indicate a significant difference.

## 3. Results

### 3.1. Clinical Information

As showed in Table 1, there were no significant differences in age and BMI among the subjects in the two groups (*p* > 0.05). In the KSD group, 42 patients (42%) had a history of urinary calculi, and 28%, 35%, and 33% patients had diabetes, hypertension, and hyperlipidemia, respectively, which were significantly higher than those in the Control group (*p* < 0.05). In addition, there were significant differences in alcohol consumption, water consumption, and diet (seafood or high fat) between patients in the KSD group and the control group (*p* < 0.05).

Further analysis of the composition of the stones in the patients in the KSD group revealed that the most abundant mixture of calcium oxalate monohydrate and dihydrate (37%; Table 2).

### 3.2. Genotypic Genetic Balance at rs13347 in the CD44 Gene

The results of HWE analysis showed that the genotype results of rs13347 locus in the CD44 gene conformed to HWE (*p* > 0.05) (Table 3), which indicated the genotype genetic equilibrium of rs13347 in the CD44 gene, and the data were derived from the same Mendel population, with the results of this test being representative.

The article "The rs13347 Polymorphism of the CD44 Gene Is Associated with the Risk of Kidney Stones Disease in the Chinese Han Population of Northeast Sichuan, China" was retracted in 2023. Reasons: signs of a paper mill; compromised peer review; unreliable results or conclusions.

### 3.3. Patients with CT and TT Genotypes at rs13347 in the CD44 Gene Were More Susceptible to Develop Kidney Stone Disease

The genotype and allele types of rs13347 in the CD44 gene were detected by PCR-RFLP in KSD and Control groups. It was found that the genotypes present in the patients were CC, CT, TT, CT+TT, and the alleles were C and T. It was also shown that patients with genotypes of CT, TT as well as CT + TT at rs13347 in the CD44 gene were more likely to have KSD. In addition to the presence of allele T at rs13347 that was also a risk factor for KSD (Table 4), which showed that the gene type at rs13347 in the CD44 gene was associated with the development of KSD.

### 3.4. Different Genotypes at rs13347 in the CD44 Gene Were Associated with the Clinical Characteristics of Patients with Kidney Stone Disease

We further compared the associations of genotypes CC, CT, and TT at rs13347 in the CD44 gene with the clinical characteristics of KSD patients, including age, BMI, recurrence or not, and so on. The results showed that the polymorphism at rs13347 in the CD44 gene was not obviously associated with age or BMI in KSD patients (*p* > 0.05), but was significantly related to whether they would relapse or not (after the first episode) and gender (*p* < 0.05). The recurrence rate of KSD was also found to be notably higher in patients with genotype CT or TT than in those with genotype CC at rs13347 in the CD44 gene (*p* < 0.05) (Table 5). Further analysis of the association between patient gender and rs13347 genotype revealed that in female patients, rs13347 polymorphism was not related to susceptibility. However, in male patients, patients with CT and TT genotypes had a prominently increased risk of KSD (Table 6). The consequences showed that polymorphism in the genotype at rs13347 in the CD44 gene was mainly associated with the risk of KSD development in male patients.

## 4. Discussion

KSD is a common disease, and it has been reported that the recurrence rate is as high as 50% within 5 years after KSD treatment [19], and patients with KSD have continued to increase over the past 50 years. Recent epidemiological data from seven countries including Italy, Japan, and the United States showed that the prevalence rate of KSD is ranging in 1.7-14.8%, and among the seven countries surveyed, the proportion is increasing [20]. The prevalence rate of KSD varies by gender, ethnicity, and geographic location. Historically, the incidence of calculus in men was two to three times higher than in women, but recent data suggest that this difference is narrowing. China is one of the highest incidence areas of KSD in the world, and KSD has become one of the most common diseases in the population of Sichuan [3]. In this study, there were 66 (66%) male KSD patients from Han population in northeast Sichuan, which is 1.94 times more than the number of female patients. Some studies have speculated that the increased prevalence rate of KSD in women may be due to lifestyle changes leading to increased obesity in women, which caused an increase in KSD patients. In addition, there were significant differences in personal habits such as alcohol consumption, water consumption, and diet (seafood or high fat) between the KSD and Control groups. Studies have confirmed a strong correlation between alcohol consumption, high-fat diet, and fish or shellfish intake and KDS prevalence [21, 22]. This is similar to our results. Other studies have pointed out that a variety of systemic diseases (diabetes, hypertension, hyperlipidemia), BMI and so on, are associated with an increased risk of KSD [23]. In the results of this research, it was found that the proportion of KSD patients with diabetes, hypertension, and hyperlipidemia symptoms was observably higher than that of the control group. However, there was no significant difference in BMI between the two groups of subjects, which was slightly different from that reported in previous studies. The difference may be due to different geographical and environmental factors at northeast area of Sichuan in China [24], or due to different local genetic differences in the population, and reports have shown that different genotypes are also the key factors inducing KSD [25].

The article "The rs13347 Polymorphism of the CD44 Gene Is Associated with the Risk of Kidney Stones Disease in the Chinese Han Population of Northeast Sichuan, China" was retracted in 2023. Reasons: signs of a paper mill; compromised peer review; unreliable results or conclusions.

The CD44 gene is encoded on the short arm of chromosome 11 in humans and is composed of 20 exons and 19 introns, with a total length of 50 kb [26]. The CD44 gene loci reported so far are rs13347, rs187115, and rs4756195, and the polymorphisms at these loci are relevant to the occurrence of tumors and related diseases of the immune system. It has been shown that CD44 is significantly highly expressed in patients with KSD [27], and it was speculated that there is a link between CD44 and the development of KSD. Studies from meta-analyses have shown a close relationship between single nucleotide polymorphisms (SNPs) and susceptibility to human disease [28]. However, due to ethnic differences [29], the role of SNPs should be investigated in different populations before they can be potentially effective biomarkers in specific genes. However, it is not clear whether SNPs in CD44 have clinical significance in KSD. In order to investigate the relationship between CD44 SNPs and the incidence of KSD of the Han population in the northeast of Sichuan Province, the genotype of the subjects was first detected by PCR-RFLP in DNA. And the SNP of rs13347 in the subjects was determined to be in HWE according to HWE analysis, indicating that the results were representative. Besides, subjects with genotypes CT and TT were found to be more likely to have KSD, which was similar to the results associated with susceptibility to induce liver cancer when nucleobase C became to T in rs13347 of CD44. In addition, it was also found that the polymorphism of rs13347 in the CD44 gene and gender are obviously related to the recurrence rate of KSD patients. That is, CT or TT genotype carrier had a significantly increased risk of KSD in male patients, and patients carrying with CT or TT were prominently associated with the recurrence rate of KSD. But in female patients, none of the polymorphisms at rs13347 were associated with susceptibility, which may be caused by the different dietary habits of women from those of men [20].

The article "The rs13347 Polymorphism of the CD44 Gene Is Associated with the Risk of Kidney Stones Disease in the Chinese Han Population of Northeast Sichuan, China" was retracted in 2023. Reasons: signs of a paper mill; compromised peer review; unreliable results or conclusions.

## 5. Conclusion

In summary, in the Han population of northeast Sichuan in China, the variant genotype (CT/TT) can increase the risk of KSD in men compared with the CD44 rs13347 CC genotype, and the CD44 gene rs13347 polymorphism may be used as a potential marker for the diagnosis and treatment of KSD. However, this study only collected the data of KSD patients in a single hospital, and it is necessary to conduct a case-control study of a wide range of populations and a carefully designed mechanistic study to verify the association between the CD44 gene polymorphism and the incidence of KSD in the Han population of northeast Sichuan, China, which was found in this trial.

## Figures and Tables

**Table 1:** General information.

	Control group (*n* = 124)	KSD group (*n* = 100)	
Age (year)	57.81 ± 11.84	58.44 ± 11.24	0.688
Male/female	93/31	66/34	N/A
BMI (kg/m^2^)	25.08 ± 4.81	24.54 ± 4.59	0.395
A history of urinary calculi (%)	N/A	42 (42%)	—
Diabetic (%)	20 (16.26%)	28 (28%)	*0.034*
Hyperpietic (%)	27 (21.95%)	35 (35%)	*0.031*
Hyperlipidemia (%)	24 (19.51%)	33 (33%)	*0.022*
Alcohol drinking (%)	27 (21.95%)	37 (37%)	*0.013*
Eat seafood (%)	21 (17.07%)	43 (43%)	*0.001*
High fat diet (%)	34 (27.64%)	47 (47%)	*0.003*
Drink water > 1000 mL/day (%)	66 (53.66%)	50 (50%)	0.587

N/A, not available. KSD: kidney stone disease.

**Table 2:** Stone composition of subjects in KSD group.

Stone composition	Number ($\underset{¯}{n}=100$)
Carbonated apatite	5
Carbonated apatite, calcium oxalate dihydrate	2
Carbonated apatite, ammonium urate	1
Carbonated apatite, calcium oxalate monohydrate	6
Carbonated apatite, calcium oxalate monohydrate and calcium oxalate dihydrate	1
70% carbonated apatite, 10% calcium oxalate monohydrate, and 20% magnesium ammonium carbonate	1
70% carbonated apatite, 20% calcium oxalate monohydrate, and 10% ammonium urate	1
Anhydrous uric acid	5
Anhydrous uric acid, calcium oxalate dihydrate	1
85% anhydrous uric acid and 15% uric acid dihydrate	1
Calcium oxalate monohydrate, calcium oxalate dihydrate	37
Carbonated apatite, calcium oxalate monohydrate, and calcium oxalate dihydrate	3
Calcium oxalate monohydrate, calcium oxalate dihydrate, and anhydrous uric acid	2
Calcium oxalate monohydrate	8
Calcium oxalate dihydrate	2
Calcium oxalate monohydrate, carbonated apatite	1
Calcium oxalate monohydrate, calcium oxalate monohydrate, and sodium urate	1
70% calcium oxalate monohydrate, 10% calcium oxalate dihydrate, and 20% carbonated apatite	6
70% calcium oxalate monohydrate, 30% calcium oxalate dihydrate	13
80% calcium oxalate monohydrate, 10% calcium oxalate dihydrate, and 10% carbonated apatite	3

KSD: kidney stone disease.

The article "The rs13347 Polymorphism of the CD44 Gene Is Associated with the Risk of Kidney Stones Disease in the Chinese Han Population of Northeast Sichuan, China" was retracted in 2023. Reasons: signs of a paper mill; compromised peer review; unreliable results or conclusions.

**Table 3:** Hardy-Weinberg equilibrium analysis of rs13347 locus in the CD44 gene.

Grouping	CC	CT	TT	C	T	HWE*χ*^2^	*p*
Control group	46	52	26	144	104	1.204	0.548
KSD group	21	47	32	89	111	0.082	0.960

**Table 4:** Genotype and allele types of rs13347 in the CD44 gene in the two groups of patients.

Genotype	Control group (*n* = 124, %)	KSD group (*n* = 100, %)	OR (95% CI)	*p*
CC	46 (37.1)	21 (21.0)	—	—
CT	52 (42.0)	47 (47.0)	1.980 (1.034-3.791)	0.038
TT	26 (21.0)	32 (32.0)	2.696 (1.298-5.559)	0.008
CT+TT	79 (63.7)	77 (77.0)	2.219 (1.213-4.057)	0.010
C	144 (58.1)	89 (44.5)	—	—
T	104 (41.9)	111 (55.5)	1.605 (1.103-2.335)	0.013

**Table 5:** Comparison of clinical characteristics of KSD patients with different genotypes of rs13347 in the CD44 gene.

	KSD patient (*n* = 100, %)			*χ* ^2^/*F*	*p*
	CC	CT	TT		
Age (year)	57.48 ± 11.38	58.68 ± 10.34	58.72 ± 12.66	0.096^b^	0.909
BMI	25.07 ± 3.84	24.50 ± 5.11	24.24 ± 4.39	0.204^b^	0.816
Gender				7.366^a^	0.025
Male	9 (13.6)	36 (54.5)	21 (31.8)		
Female	12 (35.3)	11 (32.4)	11 (32.4)		
Recurrence or not				14.524^a^	0.001
Yes	5 (8.3)	33 (55.0)	22 (36.7)		
No	16 (40.0)	14 (35.0)	10 (25.0)		

Note: a means the statistic is *χ*^2^. b means the statistic is *F*.

**Table 6:** Effect analysis between different genders and genotypes at rs13347 in the CD44 gene.

	Male		OR (95% CI)	*p*	Female		OR (95% CI)	*p*
	Control	KSD			Control	KSD		
CC	36 (38.7)	9 (13.6)	—	—	10 (32.30)	12 (35.30)	—	—
CT	41 (44.1)	36 (54.5)	3.512 (1.491-8.273)	0.004	11 (35.50)	11 (32.40)	0.833 (0.255-2.724)	0.763
TT	16 (17.2)	21 (31.8)	5.250 (1.974-13.961)	0.001	10 (32.30)	11 (32.40)	0.917 (0.276-3.040)	0.887

## Data Availability

The data used to support the findings of this study are available from the corresponding author upon request.
